# Construction of an Artificial Intelligence Writing Model for English Based on Fusion Neural Network Model

**DOI:** 10.1155/2022/1779131

**Published:** 2022-05-21

**Authors:** Meijin Hsiao, Maosheng Hung

**Affiliations:** ^1^School of Art and Design, Fuzhou University of International Studies and Trade, Fuzhou, Fujian 350202, China; ^2^School of Foreign Languages, Fuzhou University of International Studies and Trade, Fuzhou, Fujian 350202, China

## Abstract

This paper presents an in-depth study and analysis of the model of English writing using artificial intelligence algorithms of neural networks. Based on word vectors, the unsupervised disambiguation, and clustering of multimedia contexts extracted from massive online videos, the disambiguation accuracy reaches over 0.7, and the resulting small-scale multimedia context set can cover up to 90% of vocabulary learning tasks; user experiments show that the multimedia context learning system based on this method can improve the effectiveness and experience of ESL vocabulary learning, as well as the long-term word sense memory of learners. The results are 30% better. Based on the dependency grammatical relations and semantic metrics of collocations on a large-scale professional corpus, we established a collocation intention description and retrieval method in line with users' linguistic cognition and doubled the usage rate of collocation retrieval on the actual deployment system after half a year, becoming a user “sticky” ESL writing aid, and further defined style. Dictionaries only provide basic lexical definitions, and, even if supported by example sentences, they still cannot meet the needs of ESL authors in terms of expressive accuracy and richness. However, the current machine translation is based on the black box deep neural network construction, and its translation process is not understandable and interactive. Among the three algorithmic models constructed in this paper, the multitask learning model outperforms the conditional random field model and the LSTM-CRF model because the multitask learning model with auxiliary tasks solves the problem of sparse data to a certain extent, allowing the model to be trained more adequately in the case of uneven label distribution, and thus performs better than other models in the task of grammatical error detection.

## 1. Introduction

ESL writing cannot be separated from electronic text editors, and tools such as online dictionaries and automatic machine translation are currently the main tools to assist ESL writing. However, dictionaries only provide basic vocabulary definitions, and even if they are supported by example sentences, they still cannot meet the needs of ESL writers in terms of accuracy and richness of expression [1]. The current machine translation is built based on a deep neural network of a black box, and its translation process does not have comprehensibility and interactivity, nor can it effectively assist the deep cognitive thinking process in ESL writing. Therefore, in terms of application, the existing writing assistance methods are still far from the demand for high-quality and efficient writing [2]. It provides ideas and methods for the computational representation of semantics, making it possible to develop writing aids oriented to semantics and user intent. Due to the complexity of human language and writing cognition, only relying on machine automation methods cannot meet the needs of ESL high-quality writing expression. Due to the complexity of human language and writing cognition, relying on machine automation alone cannot meet the demand for high-quality writing expressions in ESL, and there is a need to study human-machine collaborative methods for aiding writing expressions by enhancing ESL's linguistic ability and to combine human intelligence and machine intelligence to solve problems.

Natural language processing (NLP) is a discipline that deals with the interaction between natural language and computers, especially the study of how to analyze huge amounts of natural language data through computer programming. Grammatical error autocorrection (GEC) is a downstream task of natural language processing that aims to automatically correct grammatical errors contained in English texts using computer-written programs [3]. An ideal GEC model should be able to detect and correct all types of grammatical errors in the input text and output a grammatically correct text that matches the original semantics expressed by the input text [4]. This is achieved using techniques and methods related to natural language processing. The automatic correction model for grammatical errors in English texts can help English teachers to correct their compositions and greatly reduce their workload, thus saving more time and energy for improving the quality of teaching. For English learners, they can get timely and effective feedback after submitting their compositions, which can improve their learning efficiency and independent learning ability. For the whole education system, it makes up for the shortage of teachers and helps to improve the education level positively. Therefore, it is of great importance to study the model of automatic correction of grammatical errors in English texts. The short textbook is a kind of text format data commonly found on the Internet [5]. In today's information age, there are countless short messages of various kinds, including cell phone text messages, spam emails, question and answer and recommendation system messages, and product reviews from shopping platforms. Extracting the information needed by humans from the short text database in a timely and accurate manner is a major challenge in the field of text classification at present.

This method uses NLP technology to analyze the text of student answers and standard answers and determine whether the answer is correct or not based on whether the answer contains domain-specific concepts. With the continuous development of artificial intelligence, increasingly intelligent devices and systems are coming into our lives. In the field of English education, the emergence of automatic English composition correction systems has greatly eased the pressure of English teachers to correct students' English compositions, and students can use these systems to quickly improve their English writing skills. Many colleges and universities have introduced these systems to assist in teaching. The workload is greatly reduced, thereby saving more time and energy to improve the quality of teaching. For English learners, they can get timely and effective feedback after submitting their compositions, which can improve their learning efficiency and autonomous learning ability. In these systems, the computer can independently complete a comprehensive quality assessment of short English essays. Although the technology in existing automatic English composition scoring systems is mature in three aspects, grammatical accuracy, lexical complexity, and syntactic complexity, the index of coherence is missing, and the final scoring results obtained by the system cannot be considered reasonable. Therefore, it is of great significance to develop a model that can automatically analyze the quality of English text coherence.

## 2. Related Works

The entity grid is extended into a graph structure, and an entity-based unsupervised graph model is proposed, which first represents the text as a bipartite graph structure of sentences and entities, and then this bipartite graph is projected using three different ways, and when the same entity exists between sentences, an edge is created between two sentence nodes to represent the whole text as an entity graph, and the average of the entity graph is calculated. The coherence of the text is analyzed by calculating the average degree of the entity graph [6]. The entity graph model optimized embedding world knowledge based on the entity graph to capture those entities that are semantically related. A rhetorical structure theory-based discourse relation model is proposed, which focuses on the discourse relation transitions between adjacent sentences and analyzes text coherence by capturing the frequency of discourse relation transitions [7]. By fusing entity-based graphs and rhetorical structure graphs based on rhetorical relations and by mining frequent subgraphs in the fused graphs, the frequencies of frequent subgraphs are used to analyze text coherence.

A clustering-based short text classification method is proposed to deal with the shortage and sparsity of short text features by embedding knowledge-derived topics from a collection of short texts of interest using a hierarchical clustering algorithm with purity control, and experiments show that the rich representation of knowledge significantly improves the accuracy of short text classification [8]. Timely and accurately extracting the information needed by human beings from the short text database is a major problem in the field of text classification. A short textbook classification model based on recurrent neural networks and convolutional neural networks is proposed, which consists of two parts: the first part represents each short textbook as a vector form using recurrent neural network (RNN) or convolutional neural network (CNN) structures, and the second part classifies the current short textbook based on the current vector representation and the previous ones, and experiments show that adding sequence information can improve the quality of the prediction, and the performance depends on the sequence information used in the model; we propose a classifier network for predicting missing features in a given instance to overcome the feature sparsity problem, using a set of unlabeled training instances, and learn the binary classifier as a feature predictor to predict whether a particular feature occurs in a given instance, by considering the implicit co-occurrence between features to demonstrate ClassiNets and summarize word co-occurrence graphs, and, by using ClassiNet, the accuracy of short text classification tasks can be statistically significantly improved without using any external resources to find relevant features [9].

The question of higher-level writing expressions such as word organization is not about right or wrong judgments but rather whether they are close to the conventions of the target language, as reflected in the computational method of judging how frequently expressions are used in the corpus [10]. Therefore, the fact-checking system automatically validates the n-gram of the author's text in the corpus together with the alternative expressions generated by the rules and provides a set of information-integrated interfaces to assist the author in making choices [11]. The PENS and FLOW systems use bilingual parallel corpus trained translation and rephrasing models to allow users to find suitable word choices, phrases, and example sentences in Chinese directly in an English context. Aiming at professional translators, a human-machine collaborative translation model is proposed, allowing users to iteratively modify the system's recommended translation results continuously in the process of translating sentences, and the system adjusts the translation model in real time to constrain the translation results according to some of the user's inputs, which significantly improves the quality and efficiency of human-machine collaborative translation compared with the traditional model of human editing based on machine-translation results. The rule-based approach uses human-developed linguistic rules, and the algorithm flags strings that do not match the predefined rules as having grammatical errors. The statistical-based approach uses a suitable mathematical model to statistically analyze the existing data samples and then sets a threshold to judge the accuracy of the strings. The machine learning-based approach is to first construct a model and then train the model with a dataset and finally use the model to predict the results.

## 3. Analytical Design of English Writing Neural Network Algorithm

In the probabilistic model of text representation, it is assumed that there is a sufficiently large ideal text corpus document set and a string used by the user for query so that the query processing can be regarded as processing the attributes of the ideal result document set. Some attributes of the documents cannot be obtained exactly, because some feature attributes are fuzzy and invisible at the time of retrieval and contribute differently to the importance of the task [12]. Therefore, the probability values of these attributes need to be estimated at the early stage of the query to determine the importance of the processing task. The estimation at the early stage of the query can return an idealized result for the desired set of documents for the query and obtain an initialized probabilistic valuation description. The probability value of these attributes needs to be estimated in the early stage of the query to determine the importance of the processing task. The estimation in the early stage of the query can return an idealized result for the document set required by the query and obtain an initial probability estimation description. The probabilistic model implemented probabilistic ranking, where, given the user's desired retrieval *Q*, the probability of retrieval is defined as *P*(*R|D*, *Q*) by ranking all documents probabilities from largest to smallest, where *R* represents the documents associated with the desired retrieval *Q*. On the contrary, *R*′ is used to represent that the document is not relevant to the desired retrieval *Q* and *P*(*R|D*, *Q*)+*P*(*R*′*|D*, *Q*)=1; that is, the relevance of the retrieval is determined using the probability binary form.

The feature vector *d*_*i*_=(*w*_*i*_^1^, *w*_*i*_^2^, *w*_*i*_^3^,…, *w*_*i*_^*n*^) represents document *D* and the feature vector *q*_*i*_=(*w*_*i*_^1^, *w*_*i*_^2^, *w*_*i*_^3^,…, *w*_*i*_^*m*^) of the required retrieval *Q*, where the weights of *d*_*i*_ and *q*_*i*_ are calculated by the binary method; that is, *w*_*i*_^1^ is defined in {0,1}, *w*_*i*_^*m*^ is defined in {0,1}, 1 represents the presence of the attribute feature, 0 represents the absence of the attribute feature, and the relevance of document *D* to the required retrieval *Q* is calculated as in the following equation:

(1) $$\begin{array}{c} P\left(R|D,Q\right)=\sum \ln\frac{p_{i}\left(1-q_{i}\right)}{q_{i}\left(1+p_{i}\right)}, \end{array}$$

where *p*_*i*_=(*r*_*i*_/*r*), *q*_*i*_=(*f*_*i*_ − *r*_*i*_/*f* − *r*), *f* is the total number of documents in all training sets, *r* is the number of documents in the document set which are relevant to the desired retrieval, *q*_*i*_ is the number of documents in the training document set containing the attribute feature *f*, and *r* represents the number of documents containing the attribute feature *f* among the *r* relevant documents.

For example, if we need to lexically label each word in a sentence and the lexical properties of each word in the sentence are in the given set of lexical properties, then the sentence can be considered as a random field. The Markov random field adds a restriction to the random field; that is, the value of a sequence in the field is only related to the value of adjacent positions and is independent of the value of other positions.

The process of algorithmically classifying the correct lexical properties for the words in a sentence is called a lexical annotation [13]. This sentence can be regarded as a random field. The Markov random field adds a restriction based on the random field; that is, the value of a certain sequence in the field is only related to the value of the adjacent position and has nothing to do with the value of other positions. The difficulty of lexical annotation varies for different languages. English words often contain multiple lexical properties, and the lexical properties of the word need to be confirmed in the contextual context, as shown in Figure 1.

Suppose that the input sequence of the model *X*={*x*_1_, *x*_2_, *x*_3_,…, *x*_*n*_}, *x*_*n*_ denotes the information input to the network at time *t*, *s*_*t*_ denotes the state of the hidden layer of the network at time *t*, *x*_*t*_ denotes the output of the network at time *t*, and the parameter matrices *U*, *V*, and *W* are the weight matrices between two adjacent moments of the input layer to the hidden layer, the hidden layer to the output layer, and the hidden layer, respectively. We use ˆy to denote the prediction result of the output layer, and $\overset{⌢}{y}$ are calculated as shown in the two following equations:

(2) $$\begin{array}{c} s_{t}=f_{\coth}\left(Ux_{t}-Ws_{t-1}\right), \end{array}$$

(3) $$\begin{array}{c} \overset{⌢}{y}=g_{\text{softmax}}\left(Vs_{t-1}\right). \end{array}$$

Semantic coherence theory, as a language theory with a wide range of content and profound meaning, has many distinctive features, and researchers have studied many aspects of it, among which the understanding of the relationship between connection and coherence is one of the most popular research directions. Firstly, the connection is a necessary condition for the text to be coherent, and the connection between sentences can be analyzed to analyze the coherence of the text. Secondly, the formation of connection in the text not only depends on the grammatical or lexical articulation mechanism in the text but also is realized in the form of semantic relationship between words and words, language rules, and so forth. In addition, connection as an important construction means, whether in the local coherence of the text or the overall coherence of the text, it has an important significance for the expression of the text content [14]. Finally, as a semantic concept, coherence has various forms of expression; it is not only linear and sequential but also hierarchical, and it is reflected not only in the microlevel of the text but also in the macrostructure of the discourse. Based on this, this paper takes semantic coherence theory as the guiding theory to analyze the coherence of the text.

In the entity graph model, the weights between the sentence nodes represent the entity information between the sentences. Except for the UP and WP projection graphs where the weights of edges are determined by the number of shared entities, in the accept projection graphs, the weights of edges are calculated based on the weights of the grammatical roles of the shared entity words in the sentences and the sentence distances, where the weights corresponding to the grammatical roles of the entity words are, respectively, 3 for the subject (S), 2 for the object (O), and 1 for the other grammatical roles (X). The weights of the grammatical roles of the entity words are 3 for the subject (S), 2 for the object (O), and 1 for the other grammatical roles (X). The specific formula for calculating the edge weights is as follows:

(4) $$\begin{array}{c} \text{Weight}\left(s_{i},s_{k}\right)=\frac{\sum_{e\in E_{ik}}w\left(e,s_{i}^{2}\right)\cdot w\left(e,s_{k}^{2}\right)}{k+i}. \end{array}$$

In the entity graph model, we use the graph feature of average degree of appearance to represent the coherence of the text. The reason for choosing the centrality measure of the average degree of output is that it allows us to evaluate the coherence of a sentence. It is because it allows us to assess how well a sentence is connected to other sentences of the text in terms of discourse entities. Secondly, the computational complexity of the mean outdegree is lower compared to other centrality metrics, maintaining the feasibility of coherence estimation on large documents and large corpora.

(5) $$\begin{array}{c} \text{AveOutDegree}\left(G\right)=\frac{1}{N}\sum_{j=1,\ldots ,N}\sum_{i=1,\ldots ,M}\text{Weight}\left(s_{i},s_{k}\right). \end{array}$$

In this paper, the subjective questions in the test corpus are classified into three major categories by topic type, definition, sequential, and general, and then into two major categories by question type, subjective questions with question words and subjective questions with question prayers. In summary, this paper classifies the subjective questions in the subjective question corpus into six categories, namely, subjective questions with question words in the defined category, subjective questions with question prayer words in the defined category, subjective questions with question words in the sequence category, subjective questions with question prayer words in the sequence category, subjective questions with question words in the general category, and subjective questions with question prayer words in the general category [15]. For different types of interrogative sentences, different subjective question marking methods were used to realize the adaptive marking of subjective questions in this paper. The details of the question classification of this paper are shown in Figure 2. The formation of connection in the text not only depends on the cohesion mechanism of grammar or vocabulary in the text but also can be realized through the semantic relationship between words, language rules, and other forms. Whether it is in the local coherence of the text or in the overall coherence of the text, it is of great significance to the expression of the text content.

The LSTM can learn the minimum time delay across more than 1000 discrete time steps by enforcing a constant error stream with a constant error conveyor within a particular cell, and the multiplicative gate cell learns to turn on and off access to the constant error stream. The LSTM is local in time and space, and its computational complexity per time step and weight is O (1). Compared with real-time recursive learning, temporal backpropagation, correlated recursive cascades, Elman networks, and neural sequence chunking, LSTM leads to more successful runs and faster learning, and LSTM can also solve complex manual long-lag tasks that previous recursive network algorithms could not solve.

Most applications require networks to contain at least three normal types of layers: input, hidden, and output. The input neuron layer can receive data from input files or directly from electronic sensors in real-time applications. The output layer sends information directly to the outside world, auxiliary computer processes, or other devices, such as mechanical control systems.

(6) $$\begin{array}{c} y=f\left(\sum_{i=1}^{n}w_{i}x_{i}+\theta \right). \end{array}$$

There can be many hidden layers between these two layers, and these inner layers contain many neurons in a variety of interconnected structures, with the inputs and outputs of each hidden neuron simply passed to the other neurons.

(7) $$\begin{array}{c} V\left(w\right)⟵V\left(w\right)-\eta \sum_{j=1}^{\ell \left(w\right)}\frac{\partial \left(w,j\right)}{\partial X_{w}^{2}}. \end{array}$$

In most networks, each neuron in a hidden layer receives signals from all neurons in the layer above it (usually the input layer), and when a neuron performs its function, it passes the output to all neurons in the layer below it, providing a feedforward path to the output. These lines of communication from one neuron to another are important aspects of neural networks; they are the glue of the system, they provide variable strength connections to the inputs, these connections are of two types, and one leads to the addition and mechanism of the next neuron, while the other leads to its subtraction, and, in more human terms, one excites, while the other inhibits as shown in Figure 3.

Finally, there is the output gate, which can determine the value of the next hidden state, which contains the relevant information from the previous input [15]. The hidden state can also be used for prediction. First, the information *h*_*t*_ − 1 of the previous hidden state and the information *X*_*t*_ of the current input are fed to the Sigmoid function; then the newly obtained cell state is passed to the Tanh function; the output of Tanh is multiplied by the output of Sigmoid, which is used to determine the information carried by the hidden state. Finally, the hidden state is output as the current unit, while the new unit state and the hidden state are passed to the next time node.

## 4. Design Analysis of English Artificial Intelligence Writing Model Construction

To estimate the duration of subjects' writing and tool use more accurately, we considered the writing process to begin when subjects first typed or switched to the tool window, thus excluding the time spent reading and understanding the task prompts [16]. The output layer sends information directly to the outside world, auxiliary computer processes, or other devices such as mechanical control systems. The average time spent by each subject on each query tool to complete each sentence as a percentage of the total writing time is shown in Figure 4. On average, subjects spent 23.5% of their total writing time on query tools, with large individual differences (minimum of 7.4%, maximum of 38.4%, and standard deviation of 9.2%). The frequency of use of each tool type is shown in Figure 4, with dictionary, Google Scholar, Google Machine Translation, and Google Web Search in descending order, and the frequency of use is positively correlated with the time spent. In addition, bilingual dictionaries were still the most relied on by the subjects: all subjects used dictionaries at least once, and nine subjects indicated that the tool use strategy was dictionary first, and three of them used dictionaries almost exclusively. This is because dictionaries have more comprehensive information and contain a variety of information such as Chinese-English translations and example sentences.

The encoder encodes the input English text sequence as an intermediate semantic vector, and the decoder decodes the intermediate semantic vector starting from the starting symbols. After the decoder generates the final probability distribution, it can correspondingly get the probability of each word in the vocabulary at the current moment and select the output of the current moment according to the output probability and using certain decoding strategies, which is an inference process of the coder and repeats until it encounters the end of the sentence indicating EOS or reaches the predefined maximum sentence length [17]. The output of each moment in the decoder is used as the input of the next moment, so the choice of decoding strategy is crucial, which directly affects the accuracy of the output results of all the later moments.

The cluster search algorithm is a heuristic graph search algorithm, which explores the graph by expanding the best nodes in a finite set, keeping only the most promising nodes, and clipping the poor-quality ones; the smaller the bundle width, the more nodes are clipped, which can improve the time efficiency and reduce the space consumption at the same time when the solution space of the graph is relatively large. However, the cluster search expands the best candidate nodes by the scores of all the previous words, which leads to the overweighting of the parent nodes, and when we expand the last K nodes, we find that the subsequent nodes of the first best node are far better than the subsequent nodes of all the other nodes, and this progenitor advantage will keep accumulating in the process of continuous expansion, resulting in the final candidate signal mainly from a single beam, with minor variations in the tails, which is also a limitation of the cluster search algorithm [18].

Because entity words appear mainly as nouns or pronouns in English texts, the accuracy of our lexical annotation results is very important for recognition results when entity words are identified. In the preprocessing module, we have used a lexical annotator with relatively good accuracy to annotate the text. Based on the lexical annotation results, we can extract the nouns and pronouns in the text. This is an inference process by the codec, and it is repeated until the end of the sentence is encountered representing EOS or the preset maximum sentence length is reached. The output of each moment in the decoder is used as the input of the next moment, so the choice of decoding strategy is very important. However, in some English texts, sometimes words such as numbers and symbols are also labeled as nouns, but they are not useful for text coherence analysis and become noise factors. So, after extracting all the entity words, this model will also filter the entity words set to reduce the noise factor, as shown in Figure 5.

However, when the VF2 subgraph matching algorithm is used for subgraph mining of the sentence semantic graph, we find that the condition for the VF2 algorithm to end the recursive method is that the number of nodes in the current set of matched states is equal to the number of nodes in the query graph that needs to be queried, which simply means that the principle of the VF2 algorithm is that once a subgraph state that fully satisfies the condition is found, the result is immediately returned and the search is ended by jumping out of the loop [19]. First, we define a set and deposit the candidate node pairs that satisfy the conditions in the feasibility judgment between the candidate node pairs and the initial matching state for the first time and then traverse the set according to the candidate node pairs in the set and the current matching states. When the subgraph state satisfies the condition, the result is saved and iterated through the other candidate node pairs until the whole set is traversed, so that we can search all the subgraphs in the target graph which are isomorphic to the query graph.

## 5. Analysis of the Results

### 5.1. Performance Results of Artificial Intelligence Neural Network Algorithm

To verify whether the improved function works better than the traditional function, the experiments will be compared in terms of both accuracy and training time, and, to make the results more accurate and to observe the effect on different classifiers, the experiments are conducted on SVM (support vector basis) and KNN (K-nearest neighbor classifier, *K* = 10) classifiers for short text classification, respectively.

The successor nodes of the first best node are far superior to the successor nodes of all other nodes. In the process of continuous expansion, this parental advantage will continue to accumulate, resulting in the generation of the final candidate signal mainly from a single beam. Minor changes can also be the limitation of the beam search algorithm. As can be seen from Figure 6, when the dimensionality is lower than 4000, the accuracy of both models decreases sharply, which is due to the removal of many important features during feature selection. When the dimension is higher than 4000, the accuracy still increases but tends to be flat. When the features are in 10,000–60,000 dimensions, the accuracy fluctuates but the fluctuations are lower, and the range of change is not large because there are redundant features when the number of features is relatively large to reach tens of thousands of dimensions, and removing some redundant features in the appropriate range can improve the efficiency of computing while having little impact on the accuracy. In both SVM and KNN, when the number of dimensions is lower than 4000, the time variation is not too big.

When the dimensionality is higher than 4000, the time of both models increases sharply, which is due to the increasing number of feature dimensions, which generates many redundant features and thus increases the classification time. From Figure 6, it is shown that, regardless of the SVM classifier or KNN classifier, the improved feature selection model sometimes has a longer training time than the traditional model, but, combined with the accuracy corresponding to the dimensions where the improved feature selection model has a longer training time than the traditional model, the improved feature selection model is more accurate than the traditional model in both cases, so it is acceptable to sacrifice some training time appropriately based on improving the accuracy. Removing some redundant features in an appropriate range can improve the computational efficiency but has little effect on the accuracy. Whether in SVM or KNN, when the dimension is lower than 4000, the time change is not too big. Therefore, it is acceptable to sacrifice some training time to improve the accuracy.

When the training set data varies from 1% to 10%, the accuracy of the proposed method is higher and is between 85 and 99%, with little fluctuation. Attention-LSTM performs poorly, with accuracy fluctuating between 40% and 90%; this is because the model Attention-LSTM achieves text serialization and incorporates an attention mechanism to distinguish text features with different weight sizes.

Since the one-way LSTM only has the semantic information below and lacks the semantic information above, when the training data is small, the text vector features represent high-dimensional sparsity and the model learning ability is poor. However, the above two models still have some influence on the classification performance when the text feature redundancy is small in the training dataset, which may lead to classification errors, and the model tends to be stable when the perturbation is added to the word embedding part of the input layer for adversarial training during the training process, as shown in Figure 7.

Most of the frequent subgraphs have a relatively large difference in the frequency of occurrence between the two types of test texts, and they can distinguish the text with good coherence from the text with poor coherence. The accuracy rate is above 90%, and the model performance is better; meanwhile the accuracy rate of the model Attention-BiLSTM varies between 70% and 95%, and the variation range is large; the performance of the model Attention-LSTM is poor, and the accuracy rate fluctuates. The larger is between 40% and 90%. If they are placed in the frequent subgraphs, they will affect the frequency distribution of the frequent subgraphs, so we filter out these subgraphs and keep those with good performance accordingly. In this way, we further filter all the frequent subgraphs mined by the VF2 algorithm, and, finally, we get the set of frequent subgraphs that can effectively capture the coherent patterns in the text, and the subsequent experiments also show that the filtered frequent subgraphs are more effective.

### 5.2. Analysis of the Experimental Results of Applying the English Intelligent Writing Model

The subjects' evaluation of the effectiveness of learning various aspects of the language is shown in Figure 8. The statistical test shows that Vivo is significantly more effective than the dictionary in learning all aspects of vocabulary knowledge. The advantage of Vivo over dictionaries lies not only in the memorization of new words but also in the knowledge of various aspects of vocabulary use. This is reflected in a better understanding of word meanings, as well as knowledge of authentic pronunciation, the use of related phrases and collocations in sentences, the emotional expressions of words, and the appropriate context of use.

The accuracy of the initial feature set on the L1 versus ESL text classification task was used as an evaluation of feature quality. We focus on the performance of the initial feature set at different textual granularities, including the whole-article level and the text-paragraph level consisting of 100, 50, and 10 sentences, respectively, where the style label of the next paragraph (i.e., whether the author of the article is ESL or not) is consistent with the style label of the article in which it is located. All features were normalized to a value between 0 and 1 based on the number of sentences and sentence length of the test text.

ESL style was used as a positive example for classification because the task of this study is concerned with the problem of identifying ESL style relative to L1 texts. We use a linear, L2 regularized SVM classifier for text style classification. Since we want the classifier to both detect most style problems and reduce false positives, we adjust the hyperparameters of the model according to the F1 values.

Unlike removing features with lower weights in SVM, the feature clustering and screening process will inevitably lead to a decrease in classification accuracy. However, since the goal of this study is not to optimize the style classification task, we need to distinguish between classification accuracy and interpretability. Despite the degraded performance in the classification task, the streamlined feature set allows authors to trace back to the text corresponding to the triggering style problem, thus providing actionable guidance suggestions for improving ESL writing style, as shown in Figure 9.

The probability estimates from the logistic regression model were used as the final style authenticity metric. Compared to SVM, the logistic regression model achieves close performance in style classification, and the predictions have probabilistic interpretation. The metric ranges from 0 to 1, with a higher value representing an L1 writing style, and vice versa. We map style metrics to a bipolar color axis to make it easier for users to understand writing style tendencies. The cross-validation results show that the accuracy and recall of the logistic regression model are higher than 70% in the worst-case scenario with a sample length of 10 sentences. We obtain multiple logistic regression models for each of the five selected features and train them simultaneously and use the predicted output of the models as a measure of the writing style of the user's text across the five categories of features and overall, with a range from 0 to 1, with higher values indicating closer to L1 writing style and vice versa. We mapped the style metric to the bipolar color axis to facilitate users' understanding of writing style tendencies.

## 6. Conclusion

The size of the manually annotated training set used in this study is quite limited for a neural network model and needs to be continuously expanded. The addition of sentences manually annotated by teachers to the training set proposed in this study is also a way to expand the dataset, but it requires the system to be used on a large scale for a long time before more data can be collected. In addition, data augmentation techniques, such as the fluency enhancement learning technique proposed by Microsoft, can also be used. On top of detecting the type of grammatical errors, there is at the same time the ability to directly correct the errors and give suggestions for correct sentences. The formation of connection in the text not only depends on the cohesion mechanism of grammar or vocabulary in the text but also can be realized through the semantic relationship between words, language rules, and other forms. Whether it is in the local coherence of the text or in the overall coherence of the text, it is of great significance to the expression of the text content. For beginners learning English, it would be helpful for learners to be able to detect grammatical errors while giving correct grammatical references, allowing them to learn independently without teacher tutoring. In the future, the end-to-end sequence model can be applied to the task of grammar error correction using the idea of machine translation to achieve the goal. The BiLSTM layer extracts information somaticized at different distances from the context, and the attention mechanism layer transforms the data encoded by the BiLSTM layer to enhance the learning task of the sequence. The model optimization layer uses the SoftMax function to minimize the error loss and classify the short text corpus; experiments are conducted on the dataset (DBpedia), and this multilayer deep learning model has better classification performance compared with the models Attention-LSTM, Attention-BiLSTM, and CNN-LSTM, which have better classification performance.

## Figures and Tables

**Figure 1:** Writing cognitive model.

**Figure 2:** Bipartite graph representation of text.

**Figure 3:** Distribution of the duration of the writing process.

**Figure 4:** Subjective evaluation of learning methods.

**Figure 5:** Flow chart of grammatical role annotation module.

**Figure 6:** Accuracy of the improved feature selection model and the traditional model on KNN.

**Figure 7:** Change of writing evaluation value.

**Figure 8:** The most frequent features mentioned by subjects to distinguish L1 from ESL writing styles.

**Figure 9:** 5-Fold cross-validation results for different feature subsets on a text classification task of 100 sentences in length.

## Data Availability

The data used to support the findings of this study are available from the corresponding author upon request.
